RETRACTED

# MicroRNA-139-5p inhibits cell viability, migration and invasion and suppresses tumor growth by targeting HDGF in non-small cell lung cancer

**DOI:** 10.3892/ol.2020.11296

**Published:** 2020-01-13

**Authors:** Zuxiong Zhang, Weizhi Li, Damei Jiang, Chi Liu, Zhenghong Lai

**Affiliations:** 1 Department of Cardiothoracic Surgery, First Affiliated Hospital of Gannan Medical University, Ganzhou, Jiangxi 341000, P.R. China; 2 Department of Radiotherapy, Tumor Hospital of Ganzhou, Ganzhou, Jiangxi 341000, P.R. China; 3 Department of Obstetrics and Gynecology, Ganzhou Municipal Hospital, Ganzhou, Jiangxi 341000, P.R. China; 4 School of Medical and Life Sciences, Chengdu University of TCM, Chengdu, Sichuan 610072, P.R. China

**Keywords:** microRNA-139-5p, apoptosis, metastasis, hepatoma-derived growth factor, non-small cell lung cancer

## Abstract

MicroRNA (miRNAs) serve key roles in the progress of various types of cancer. The expression of miRNA (miR)-139-5p is downregulated in several types of tumor and has been recognized as a tumor suppressor. However, the role of miR-139-5p in non-small cell lung cancer (NSCLC) has not been investigated in detail. In the present study, it was demonstrated that miR-139-5p was significantly downregulated in NSCLC cells and tissues, and the overexpression of miR-139-5p *in vitro* induced apoptosis and significantly inhibited the viability and proliferation of A549 and H1299 cells. In addition, upregulation of miR-139-5p significantly inhibited the migration and invasion of A549 and H1299 cells. Hepatoma-derived growth factor (HDGF) was identified as a direct target of miR-139-5p. Rescue experiments demonstrated that the inhibitory function of miR-139-5p on cell viability, migration and invasion was partially mediated by suppressing HDGF expression. Furthermore, miR-139-5p exhibited efficient inhibition of tumor growth in a xenograft tumor mouse model of A549 cells. In summary, the results from the present study suggested that miR-139-5p may serve an important role in NSCLC by targeting HDGF and causing inhibition of cell viability and metastasis, as well as induction of apoptosis. miR-139-5p may also have the potential to serve as a therapeutic target for the treatment of NSCLC.

## Introduction

Lung cancer is the main cause of cancer-associated mortality worldwide, and ~85% of all lung cancer cases are classified as non-small cell lung cancer (NSCLC) by histopathological analysis (1). Despite recent advances in cancer therapy, the 5-year survival rate of patients with NSCLC remains to be just 16% (2). The development of lung cancer is a multistep process, which requires the contribution of numerous oncogenes and tumor suppressors (3–5). However, the underlying mechanism of NSCLC development remains unknown. Therefore, an improved and deeper understanding of the detailed mechanisms of NSCLC progression may be useful for the identification of new therapeutic targets and the development of novel strategies for the treatment of NSCLC.

RETRACTED

MicroRNAs (miRNAs) are small non-coding RNAs that bind to the complimentary recognition sequences of the 3′-untranslated region (3′-UTR) of target mRNAs and lead to their degradation. This process suppresses the mRNA molecules from being translated into protein molecules (6–8). miRNAs serve as a regulator for the expression of a wide variety of target genes that are involved in several biological processes, including cell proliferation, differentiation, migration and apoptosis (9–12). The deregulation of the miRNA expression levels has been suggested to be crucial in tumorigenesis and cancer progression (13,14). miRNA (miR)-139-5p has been identified as a tumor-suppressing miRNA owing to its downregulation in several types of cancer, such as gastric, breast and colorectal cancer (15). Upregulation of miR-139-5p resulted in an increase in cancer cell apoptosis *in vitro* (16). However, the detailed role of miR-139-5p in NSCLC remains poorly understood.

Hepatoma-derived growth factor (HDGF) is a heparin-binding growth factor that is involved in angiogenesis (17). The overexpression of HDGF is related with poor clinical outcomes of patients with several types of cancer. For example, the expression of HDGF is associated with poor prognosis in patients with hepatocellular carcinoma, and with poor disease-free survival and overall survival (OS) in patients with gastric carcinoma (18,19). HDGF overexpression has been demonstrated in NSCLC *in vitro* and *in vivo*, and was associated with a high probability of tumor relapse and distant metastasis (20).

In the present study, it was demonstrated that miR-139-5p expression was significantly downregulated in NSCLC, whereas overexpression of miR139-5p significantly inhibited NSCLC cell viability and migration. Furthermore, HDGF was identified as a target gene of miR-139-5p and it was suggested that miR-139-5p may inhibit tumor progression by downregulating HDGF.

## Materials and methods

### 

#### Cell lines and patient samples

Three NSCLC cell lines (A549, H1299 and Calu3) and one normal bronchial epithelial cell line (16HBE) were purchased from the Institute of Biochemistry and Cell Biology of the Chinese Academy of Sciences (Shanghai, China). The cells were cultured in DMEM containing 10% FBS, 100 U/ml penicillin and 100 mg/ml streptomycin (Invitrogen; Thermo Fisher Scientific, Inc.) in a humidified atmosphere at 37°C with 5% CO_2_.

RETRACTED

Paired NSCLC and adjacent non-tumor lung tissues (~4 mm away from the tumor) were obtained from 30 patients (male, n=17; female, n=13), who underwent surgery without radiotherapy, chemotherapy or any other therapies at the First Affiliated Hospital of Gannan Medical University (Ganzhou, China). The patients' ages ranged from 37–79 years (≥60, n=12; <60, n=18; mean age, 58.88±12.65 years). The present study was approved by the Ethics Review Committee of the First Affiliated Hospital of Gannan Medical University, and written informed consent was obtained from all patients. A 48-month follow up survival survey, based on patient medical documents was performed. OS was defined as the interval between resection and mortality, or the last follow-up visit. Pathological evaluations of the tissues were performed by pathologists from the Department of Pathology at the First Affiliated Hospital of the Gannan Medical University. The obtained tissues were stored at −80°C for further use.

#### Quantitative reverse transcription-quantitative PCR (RT-qPCR)

Total RNA was extracted from tumor tissue samples (~3.0 g) or cells (1×10^7^) using the TRIzol^®^ reagent (Invitrogen; Thermo Fisher Scientific, Inc.) according to the manufacturer's instructions. RT was conducted in order to convert RNA into cDNA using a reverse transcription kit (Thermo Fisher Scientific, Inc.) at 55°C for 45 min. qPCR was performed using an IQ SYBR-Green Supermix on the iCycler IQ multi-color detection system (both from Bio-Rad Technologies, Inc.). The thermocycling conditions for PCR were as follows: Stage 1, 95°C for 30 sec (1 cycle); stage 2, 95°C for 5 sec and 60°C for 34 sec (40 cycles); stage 3, dissociation. Stem-loop primers were used to detect miRNAs and were obtained from Guangzhou RiboBio Co., Ltd. The expression levels of the housekeeping genes U6 and GAPDH were used to normalize the expression levels of the genes of interest. The relative expression levels of each gene of interest were calculated and normalized using the 2^−ΔΔCq^ method (21) and Bio-Rad CFX manager software (version 3.1; Bio-Rad Technologies, Inc.). The primer sequences used were as follows: miR-139-5p RT primer (stem-loop), 5′-GTCAGAAGGAATGATGCACAGCCACTGGAG-3′; forward miR-139-5p, 5′-TCTACAGTGCACGTGTCTCCAG-3′; miR-139-5p reverse, 5′-ACCTGCGTAGGTAGTTTCATGT-3′; GAPDH forward, 5′-TCTCTGCTCCTCCTGTTC-3′; GAPDH reverse, 5′-GGTTGAGCACAGGGTACTTTATTGA-3′.

#### Transfection

Hsa-miR-139-5p mimic, hsa-miR-139-5p mimic negative control (miR-NC), pcDNA3-HDGF and pcDNA3-plasmid control vector were purchased from Guangzhou RiboBio Co., Ltd. For convenience, pcDNA3-HDGF and pcDNA3-plasmid control vector were referred to as HDGF and empty vector, respectively. The cells were cultured in complete DMEM medium without antibiotics for 24 h and subsequently washed with PBS (pH 7.4). The cells were transfected with 2 µg of miR-139-5p mimic, miR-NC, HDGF overexpression or empty vectors using Lipofectamine^®^ 2,000 (Invitrogen; Thermo Fisher Scientific, Inc.) according to the manufacturer's instructions. Following 48 h post-transfection at 37°C, the transfected cells were collected for further use.

RETRACTED

#### Cell viability and colony-formation assay

Cell viability was determined using the MTT cell viability assay kit (Roche Applied Science). The cells were cultured in 96-well microtiter plates at a density of 4,000 cells/well. Following treatment for 48 h, the cells were incubated with 20 µl of MTT (5 mg/ml) in culture medium for 3 h. Subsequently, 150 µl of DMSO was added into each well to dissolve the precipitated formazan, and the absorbance was measured at 570 nm. All experiments were performed in triplicate. The data were expressed as mean ± SD.

The cells that were transfected with different plasmids were collected and seeded in 6-well plates at a density of 500 cells/well. Following attachment, the cells were incubated for 6–8 days. Finally, the cells were washed with PBS, fixed with methanol for 10 min and stained with 0.1% crystal violet at 37°C for 30 min. The analysis of the cells was performed with imaging by a light microscope (Olympus Corporation; magnification, ×4).

#### Cell apoptosis assay

Cells were seeded (2×10^5^ cells/well) in 6-well plates, transfected with miR-139-5p or miR-NC for 48 h and analyzed using the Annexin V-FITC/PI cell apoptosis detection kit (Nanjing KeyGen Biotech Co., Ltd.). A total of 2×10^5^ cells were collected, suspended in 400 µl of 1X binding buffer and incubated with 5 µl of Annexin V-FITC and 5 µl of propidium iodide in the dark at room temperature for 15 min. Finally, the cells were analyzed by flow cytometry (FACScan^®^; BD Biosciences) using the FACSuit software (version: 2016; supplier: BD Biosciences).

#### Wound healing assay

Following incubation at 37°C for 24 h, the cell cultures of ~90% confluence were scratched with a 10-µl pipette tip. The floating cells were removed by washing with PBS and the attached cells were transfected with miR-139-5p and miR-NC. The incubation was performed at 37°C for another 24 h in cultured medium with 1% FBS and the cells were imaged with a light microscope (Olympus Corporation; magnification, ×4) for motility analysis. The relative migration rate was calculated as: (d1-d2)/d1 × 100%; where d1 was the width between the two edges of the wound at 0 h, and d2 was the width between two edges of the wound at 24 h.

RETRACTED

#### Migration and invasion assay

Following transfections, the cells were harvested and washed once with PBS (pH 7.4) for further use. For cell migration evaluation, 8-mm pore size culture Transwell inserts (Costar; Corning Inc.) were placed into the wells of 24-well culture plates, separating the upper and lower chambers. In the upper chamber, 5×10^4^ cells, which were suspended in 300 µl of serum-free medium, were added, and 500 µl of cultured medium containing 10% FBS was added to the lower chamber. For the Matrigel invasion assay, 1×10^5^ cells were added into the upper chamber, which were pre-coated with Matrigel. The cultures were incubated for 24 h at 37°C, and the non-migrated and non-invasive cells located on the upper surface of the filter were removed with a cotton swab, whereas the migrated and invasive cells on the bottom surface of the membrane were fixed with methanol and stained with 0.1% crystal violet at 25°C for 30 min. Finally, the cells were visualized using a light microscope (Olympus Corporation; magnification, ×100), and their number was estimated by manual counting.

#### Western blot analysis

Western blot analysis was performed to determine the change in the expression levels of the target proteins examined. The total cellular proteins were obtained from cultured cells with lysis buffer (20 mM Tris pH 7.4, 150 mM NaCl, 5 mM EDTA, 50 mM NaF and 0.1% NP-40). Total protein extracts (20 µg) were separated SDS-PAGE on a 10% gel and transferred to PVDF membranes. The membranes were blocked with 5% skimmed milk for 2 h at room temperature and incubated with primary antibodies against cleaved caspase-3 (cat. no. 9664), Bcl-2 (cat. no. 15071), matrix metalloproteinase (MMP)-9 (cat. no. 13667), MMP-2 (cat. no. 40994), HDGF (cat. no. 52445) and β-actin (cat. no. 3,700) (all 1:1,000; all from CST Biological Reagents Co., Ltd.) at 4°C overnight. The following morning, the membranes were washed with PBS and incubated with horseradish peroxidase-labeled secondary antibodies (cat. no. 7076; host, horse; dilution, 1:10,000) for 2 h at 37°C. The protein bands were visualized and imaged using a chemiluminescence detection system (Shanghai Qinxiang Scientific Instrument Co., Ltd.).

#### Luciferase reporter assays

TargetScan (http://www.targetscan.org/vert_71/; version 7.1) was used to screen the target genes of miR-139-5p. The 3′-untranslated region (UTR) of wild-type (WT) and mutant (Mut) HDGF were amplified from human genomic DNA and individually inserted into pmiR-RB-REPORT™ luciferase vectors (OBiO Technology Corp., Ltd.). A549 (5×10^6^ cells) and H1299 (5×10^6^ cells) were co-transfected with 200 ng of Mut or WT pmiR-RB-REPORT™ plasmid and 100 ng of miR-139-5p mimics or miR-NC by Lipofectamine^®^ 2000 (Invitrogen; Thermo Fisher Scientific, Inc.) according to the manufacturer's instructions. After 48 h, cells were harvested and luciferase activity was measured using a Dual-Luciferase Reporter Assay system (Promega Corporation) according to the manufacturer's protocol. *Renilla* luciferase activity was used for normalization.

RETRACTED

#### In vivo anti-tumor assays

In the present study, 10 male Balb/c nude mice (6–8 weeks, 16–20 g) were purchased from Beijing Huakangkang Biotechnology Co., Ltd. Mice were housed under specific pathogen-free (SPF) conditions (18–29°C, 40–70% humidity, 12 h light/dark cycle) and were given ad libitum access to food and water and were quarantined for 1 week in a separate SPF room, and observed any changes in the conditions of mice (weight, hair, diet and appearance) before experiment prior to treatment. All animal procedures were conducted in accordance with the protocol approved by the Institutional Animal Care and Treatment Committee of Gannan Medical University. The health and behavior of the mice were monitored every day. All mice were treated humanely throughout the experimental period. A total of 200 µl A549 cells (1×10^7^ cells transfected with miR-139-5p or miR-NC were subcutaneously injected into the right flank of the Balb/c nude mice (n=5 mice/group) to establish a xenograft NSCLC model. A total of 7 days following the injections, the tumor volume was measured simultaneously every 4 days until day 24 using the following equation: (length × width^2^) × 0.5. The first time the tumor size was measured was defined as the 0 day. Treatment was completed when the mice in the miR-NC group became moribund (at day 24; humane endpoint of the experiment was when the maximum tumor volume was no more than 1800 mm^3^). The mice were sacrificed by performing cervical dislocation, and the tumors were collected, weighed and imaged. Finally, the tumor specimens were fixed with 4% paraformaldehyde at 25°C for 24 h for further immunohistochemical analysis.

For immunohistochemistry, the frozen 4-µm-thick sections were incubated with primary rabbit anti-mouse antibody Ki-67 (dilution, 1:400; cat. no. 9449; Cell Signaling Technology, Inc.) at 25°C for 1 h, blocked with goat serum (10% in PBS; Beyotime Institute of Biotechnology) at 25°C for 15 min and subsequently treated with biotinylated goat anti-rabbit immunoglobulin secondary antibody (dilution, 1:1,000; cat. no. ab6721; Abcam) at 37°C for 30 min. The sections were incubated with streptavidin-peroxidase and DAB solution (Beijing Solarbio Science & Technology Co., Ltd.) at 37°C for 20 min to visualize the biotinylated goat anti-rabbit immunoglobulin. The sections were then treated with hematoxylin at room temperature for 10 seconds to stain the nuclei of the tumor cells. Finally, the sections were imaged and examined under a light microscope (Olympus Corporation; magnification, ×40).

RETRACTED

#### Statistical analysis

All experiments were conducted in triplicate and the data were presented as mean ± standard deviation. The statistical analysis was conducted using SPSS software (version 17.0; SPSS, Inc.). Kaplan-Meier tests were used to assess survival time. The log-rank test was used to analyze the effect of clinical variables and miRNAs on patients' OS. The median level of miR-139-5p was used as the cutoff value. Significant differences between two groups were analyzed using a Student's t-test (parametric) or Mann-Whitney U test (non-parametric). Tukey's post-hoc test was performed following one-way ANOVA; LSD's post-hoc test was performed after repeated measures ANOVA, which was used to analyze tumor size over time. *P<0.05 was considered to indicate a statistically significant difference.

## Results

### 

#### miR-139-5p is downregulated in NSCLC cells and tissues and is associated with poor prognosis

To determine whether miR-139-5p is downregulated in lung cancer, the expression levels of miR-139-5p in human primary lung tumors (NSCLC) and pair-matched adjacent lung normal tissues were examined using RT-qPCR. The expression levels of miR-139-5p were significantly (P<0.05) reduced in the NSCLC compared with the normal tissues (Fig. 1A). The expression levels of miR-139-5p were also investigated in several NSCLC cell lines (A549, H1299 and Calu3), in which the expression levels were significantly (P<0.01) lower compared with those of the 16HBE normal lung cells (Fig. 1B). In addition, it was revealed that the downregulation of miR-139-5p was significantly (P<0.005) associated with the clinical stage (Fig. 1C). Moreover, Kaplan-Meier survival analysis further demonstrated that downregulation of miR-139-5p was associated with poor OS in patients with NSCLC (P<0.05; Fig. 1D). Overall, these results suggested that downregulation of miR-139-5p expression may be associated with poor prognosis in patients with NSCLC.

#### miR-139-5p inhibits NSCLC cell viability and induces apoptosis

To investigate the antitumoral role of miR-139-5p in NSCLC cells, miR-139-5p or miR-NC was transfected into A549 and H1299 cells. As expected, the expression levels of miR-139-5p in A549 (Fig. 2A) and H1299 (Fig. 2B) cells were significantly increased following miR-139-5p transfection compared with those transfected with miR-NC. Subsequently, the role of miR-139-5p on H1299 and A549 cell viability was evaluated. MTT assays revealed that miR-139-5p significantly (P<0.01) inhibited the viability of both A549 and H1299 cells compared with mi-NC-transfected cells at day 3 and 4 post-transfection (Fig. 2C and D, respectively). When the expression level of miR-139-5p was reduced (Fig. 2E), the colony-forming ability of 16HBE normal epithelial cells was not changed significantly (Fig. 2F). Furthermore, the results of the colony-formation assays indicated that miR-139-5p overexpression significantly suppressed the viability of A549 and H1299 cells (Fig. 2G). In addition, miR-139-5p transfection induced NSCLC cell apoptosis as demonstrated by flow cytometry. In the A549 and H1299 cell lines, miR-139-5p caused a significant increase in the number of late apoptotic cells (annexin^+^/PI^+^) compared with that in miR-NC-treated cells (Fig. 2H). The effects of miR-139-5p on the expression levels of the apoptotic proteins were investigated by western blot analysis. The expression levels of cleaved caspase-3 were notably increased, whereas the expression levels of Bcl-2 were decreased following transfection with miR-139-5p compared with miR-NC in both in A549 and H1299 cells (Fig. 2I). These results suggested that miR-139-5p inhibited viability and induced apoptosis of NSCLC cells.

RETRACTED

#### miR-139-5p suppresses NSCLC cell migration and invasion

Wound healing, Transwell and Matrigel assays were used to assess the anti-migratory and anti-invasive activities of miR-139-5p *in vitro*. Compared with miR-NC-treated group, miR-139-5p treated cells had significantly lower migration rate in both A549 and H1299 cells (Fig. 3A; P<0.001). In addition, migration (Fig. 3B) and invasion (Fig. 3C) were significantly inhibited by treatment of the A549 and H1299 cells with miR-139-5p compared with the respective miR-NC groups. Furthermore, the anti-metastatic mechanism of action was investigated by analyzing the expression levels of the apoptotic proteins via western blot analysis. The expression levels of MMP-2 and MMP-9 were notably decreased following treatment with miR-139-5p compared with those in the miR-NC group in both cell lines (Fig. 3D). Therefore, these results suggested that miR-139-5p may effectively inhibit NSCLC invasion *in vitro*.

#### miR-139-5p inhibits NSCLC cell viability, migration and invasion by targeting HDGF

To investigate the role of miR-139-5p in the progression of NSCLC, TargetScan was used to screen the target genes of miR-139-5p. HDGF is an oncogene noted in several types of cancer (22), including NSCLC, and was predicted to be a target of miR-139-5p (Fig. 4A). Luciferase activity assay demonstrated that miR-139-5p significantly suppressed the luciferase activity of the HDGF-WT 3′-UTR but not that of HDGF-Mut 3′-UTR in the A549 and the H1299 cells, compared with the respective miR-NC transfected cells (Fig. 4B). In addition, increased miR-139-5p expression in A549 and H1299 cells reduced HDGF mRNA and protein expression levels (Fig. 4C and D).

RETRACTED

Further experiments were used to investigate the interaction between HDGF and miR-139-5p. Overexpression of HDGF was established by transfection with HDGF expression vector (Fig. 4E), which resulted in significant (P<0.001) impairment of the inhibitory function of miR-139-5p on viability, migration and invasion of A549 cells (Fig. 5A-C). There were no statistically significant differences of colony formation, migration and invasion between miR-NC and miR-NC + HDGF groups. These results suggested that miR-139-5p inhibited NSCLC cell viability, migration and invasion by targeting HDGF.

#### miR-139-5p inhibits tumor growth in vivo

Balb/c nude mice were used in xenograft experiments, in which A549 cells transfected with miR-139-5p or miR-NC were subcutaneously injected to assess the tumor suppressor function of miR-139-5p. The tumor volume was measured every 4 days until day 24. The tumor volume at 24 days and tumor weight were significantly reduced in the miR-139-5p group compared with those of the miR-NC group (Fig. 6A-C). The result of the immunohistochemical analysis indicated suppressed expression levels of Ki-67 by miR-139-5p (Fig. 6D), in comparison with the miR-NC group, which suggested that miR-139-5p inhibited tumor growth *in vivo*.

## Discussion

In the present study, it was demonstrated that miR-139-5p express was significantly lower in NSCLC tissues and cell lines. It was observed that overexpression of miR-139-5p markedly inhibited the viability of NSCLC cells, and led to a concomitant induction of NSCLC cell apoptosis. Overexpression of miR-139-5p significantly induced cell apoptosis, which may have a direct effect on cell viability. Furthermore, increased miR-139-5p expression significantly suppressed the migration and invasion of NSCLC cells. Using luciferase activity and western blot assays, it was demonstrated that HDGF was a direct target of miR-139-5p. miR-139-5p inhibited cell viability and invasion by targeting HDGF. Overexpression of miR-139-5p significantly inhibited tumor growth in a xenograft tumor mouse model. Overall, the results from the present study revealed that miR-139-5p inhibited NSCLC cell viability *in vitro* and suppressed tumor growth *in vivo*.

Numerous miRNAs have been identified in NSCLC and a number of these molecules serve key roles in various biological processes, such as metastasis, viability, differentiation, apoptosis and immune responses (23,24). The deregulation of miRNAs is associated with the development of several types of disease, including cancer (25,26). Tumor-associated miRNAs can serve as oncogenes or tumor suppressors depending on whether their target is a tumor suppressor gene or an oncogene. The deregulated expression levels of specific miRNAs could affect tumor metastasis and prognosis through the regulation of numerous pathways (27). Yanaihara *et al* (7) suggested that miR-155 was upregulated in NSCLC tissues and that it was associated with poor survival of NSCLC patients. Ke *et al* demonstrated that miR-149, which was downregulated in NSCLC tissues, suppressed the epithelial-to-mesenchymal transition process of A549 cells by targeting Forkhead box M1 (14). The expression levels of miR-181b have been revealed to be associated with distant organ metastasis, and higher p-Tumor-Node-Metastasis stage of patients with NSCLC (28). miR-16 has been identified as a tumor suppressor, which inhibits cancer cell growth and proliferation *in vitro* via the insulin-like growth factor 1 receptor, the Raf1/mitogen-activated protein kinase kinase 1/2/ERK 1/2 and the p53/survivin signaling pathways (29,30). In the present study, it was demonstrated that HDGF served as a direct target of miR-139-5p, and that miR-139-5p could inhibit NSCLC cell proliferation and metastasis by suppressing HDGF expression. HDGF is upregulated in various types of cancer and is associated with increased cancer cell proliferation, angiogenesis and metastasis (17,31).

RETRACTED

In conclusion, the present study provided evidence that miR-139-5p was significantly downregulated in NSCLC cell lines and tissues. Upregulation of miR-139-5p in NSCLC cells suppressed viability, migration and invasion by inhibiting HDGF expression. These findings suggested that miR-139-5p may serve as a potential therapeutic target for the treatment of NSCLC.

## Figures and Tables

**Figure 1.** miR-139-5p expression is downregulated in NSCLC and associated with tumor progression and poor overall survival. (A) miR-139-5p expression levels in NSCLC tumor tissues and adjacent normal tissues. *P<0.05. (B) miR-139-5p expression in the NSCLC cell lines A549, H1299 and Calu3, and in the normal bronchial epithelial cell line 16HBE. *P<0.05 and **P<0.01 vs. 16HBE. (C) Relative expression levels of miR-139-5p in different stages of NSCLC tumor tissues. *P<0.05. (D) Overall survival rate based on expression levels of miR-139-5p in 30 patients with NSCLC. miR, microRNA; NSCLC, non-small cell lung cancer.

**Figure 2.** miR-139-5p inhibits NSCLC cell viability and induces apoptosis. (A and B) RT-qPCR was used to determine the expression levels of miR-139-5p in (A) A549 and (B) H1299 cells after being transfected with miR-139-5p. **P<0.01 vs. miR-NC. (C) A549 and (D) H1299 cell viability was evaluated by MTT assay following miR-139-5p transfection. **P<0.01. (E) miR-139-5p expression levels were measured by RT-qPCR following transfection with si-NC or si-miR-139-5p. (F) Change of colony formation ability of 16HBE cells treated with si-miR139-5p and si-NC. (G) Colony formation assay of A549 and H1299 cells transfected with miR-139-5p. *P<0.05 and **P<0.01 vs. miR-NC. (H) A549 and H1299 cell apoptosis was increased by miR-139-5p, as assessed using an Annexin V-FITC/PI staining flow cytometry assay. ***P<0.001 vs. miR-NC. (I) Expression levels of apoptosis associated proteins cleaved caspase 3 and Bcl2 were analyzed by western blotting. miR, microRNA; NC, negative control; NSCLC, non-small cell lung cancer; OD, optical density; PI, propidium iodide; RT-qPCR, reverse transcription-quantitative PCR.

RETRACTED

**Figure 3.** miR-139-5p inhibits NSCLC cell migration and invasion. (A) The migratory ability of transfected A549 and H1299 cells was evaluated using a wound healing assay. The edges of the wounds are marked with white lines. (B) Migratory and (C) invasive abilities of transfected A549 and H1299 cells were evaluated by Transwell and Matrigel assays, respectively. **P<0.01 and ***P<0.001 vs. miR-NC. (D) Expression levels of metastasis-associated proteins MMP-9 and MMP-2 were analyzed by western blotting. miR, microRNA; NC, negative control; NSCLC, non-small cell lung cancer; MMP, matrix metalloproteinase.

**Figure 4.** HDGF is a direct target of miR-139-5p. (A) Predicted binding sites between HDGF and miR-139-5p. (B) Luciferase activity in A549 and H1299 cells co-transfected with miR-139-5p or miR-NC and HDGF-WT or HDGF-Mut. (C) RT-qPCR analysis of the relative mRNA expression levels of HDGF in A549 and H1299 cells transfected with miR-139-5p or miR-NC. (D) Western blot analysis of HDGF protein expression in transfected A549 and H1299 cells. (E) mRNA expression levels of HDGF were measured by RT-qPCR in untransfected Control cells and those transfected with empty vector and HDGF overexpression vector. *P<0.05, **P<0.01 and ***P<0.001. HDGF, hepatoma-derived growth factor; miR, microRNA; Mut, mutant; RT-qPCR, reverse transcription-quantitative PCR; WT, wild-type.

**Figure 5.** miR-139-5p inhibits A549 non-small cell lung cancer colony formation, migration and invasion by suppressing expression of HDGF. (A) Colony formation ability in A549 cells. (B) Migration and (C) invasion abilities of transfected A549 cells evaluated by Transwell and Matrigel assays, respectively. ***P<0.001 vs. miR-NC. HDGF, hepatoma-derived growth factor; miR, microRNA; NC, negative control.

RETRACTED

**Figure 6.** miR-139-5p suppresses tumor growth *in vivo*. (A) Representative images of tumors from miR-139-5p and miR-NC xenografted mice at day 24. (B) Growth curve drawn by measuring tumor volumes at the indicated times. (C) Tumor weight of miR-139-5p and miR-NC groups at day 24. (D) Evaluation of Ki-67 in tumor section of miR-139-5p and miR-NC groups. **P<0.01. miR, microRNA; NC, negative control.

## Data Availability

The datasets used and/or analyzed during the present study are available from the corresponding author upon reasonable request.
